# Hormone Replacement Therapy and Aging: A Potential Therapeutic Approach for Age-Related Oxidative Stress and Cardiac Remodeling

**DOI:** 10.1155/2021/8364297

**Published:** 2021-02-03

**Authors:** Renáta Szabó, Alexandra Hoffmann, Denise Börzsei, Krisztina Kupai, Médea Veszelka, Anikó Magyariné Berkó, Imre Pávó, Rudolf Gesztelyi, Béla Juhász, Zsolt Turcsán, Anikó Pósa, Csaba Varga

**Affiliations:** ^1^Department of Physiology, Anatomy and Neuroscience, Faculty of Science and Informatics, University of Szeged, Szeged H-6726, Hungary; ^2^Interdisciplinary Excellence Centre, Department of Physiology, Anatomy and Neuroscience, University of Szeged, Szeged, Hungary; ^3^1st Department of Medicine, University of Szeged, Szeged H-6720, Hungary; ^4^Department of Pharmacology and Pharmacotherapy, University of Debrecen, Debrecen H-4032, Hungary

## Abstract

Advanced age is an independent risk factor for cardiovascular diseases, which might be further exacerbated by estrogen deficiency. Hormone replacement therapy (HRT) decreases cardiovascular risks and events in postmenopausal women; however, its effects are not fully elucidated in older individuals. Thus, the aim of our study is to examine the impact of HRT on oxidant/antioxidant homeostasis and cardiac remodeling. In our experiment, control (fertile) and aging (~20-month-old) female Wistar rats were used. Aging rats were further divided into estrogen- (E_2_, 0.1 mg/kg/day *per os*) or raloxifene- (RAL, 1.0 mg/kg/day *per os*) treated subgroups. After 2 weeks of treatment, cardiac heme oxygenase (HO) activity, total glutathione (GSH) content, matrix metalloproteinase-2 (MMP-2) activity, and the concentrations of collagen type I and tissue inhibitor of metalloproteinase (TIMP-2), as well as the infarct size, were determined. The aging process significantly decreased the antioxidant HO activity and GSH content, altered the MMP-2/TIMP-2 signaling, and resulted in an excessive collagen accumulation, which culminated in cardiovascular injury. However, 2 weeks of either E_2_ or RAL treatment enhanced the antioxidant defense mechanisms and attenuated cardiac remodeling related to aging. Our findings clearly show that 2-week-long HRT is a potential intervention to bias successful cardiovascular aging via reducing oxidative damage and cardiovascular dysfunction.

## 1. Introduction

Cardiac senescence is characterized by morphological and functional changes that render the heart and vasculature to be prone to cardiovascular diseases (CVDs). Although the mechanisms underlying cardiovascular aging are complex and involve multiple pathways, a growing body of evidence shows that chronic oxidative stress is a key factor in the incidence and progression of CVDs [1–3].

High levels of reactive oxygen species (ROS) may play a critical role in the cellular damage during aging and lead to an imbalance between the oxidant and antioxidant systems [4]. Shift in the redox status can result from disturbances in the antioxidant defense systems, including superoxide dismutases, glutathione peroxidase, catalase, peroxiredoxin, and nonenzymatic antioxidants, such as glutathione (GSH) [5]. Age-related GSH depletion is associated with ROS overproduction and makes the heart more vulnerable to macromolecular damage affecting the physiological mechanisms and function [6]. Additional ROS-sensitive defense mechanisms involve the heme oxygenase (HO) enzyme system that provides an adaptive cellular response against oxidative injury and chronic inflammation by the conversion of heme to the metabolites carbon monoxide (CO), free iron, and biliverdin [7]. Besides its antioxidant and anti-inflammatory properties, increased activity of HO ameliorates left ventricular dysfunction, hypertrophy, and interstitial fibrosis and improves tissue neovascularization with a great impact on cardiac remodeling processes [8]. Due to the impaired endogenous defense systems and increased production of ROS, oxidative stress-induced pathways lead to maladaptive fibrotic processes in the myocardium, thus promoting the development of pathological cardiac remodeling. Age-associated cardiomyocyte loss and excessive collagen deposition (i.e., fibrosis) result in the critical deterioration of the extracellular matrix [9].

Numerous studies suggest that both oxidative and fibrotic changes can be associated with the altered action of estrogen via estrogen receptors. Estrogen binds to traditional estrogen receptor alpha (ER*α*) and estrogen receptor beta (ER*β*), expressed in vascular endothelial cells, vascular smooth muscle cells, and cardiomyocytes, thus playing an important role in maintaining vascular tone, oxidant/antioxidant balance, and antifibrotic effects under healthy conditions [10]. While estrogen exerts antioxidative, vasodilatory, and antifibrotic effects, aging-mediated estrogen depletion increases mitochondrial dysfunction and oxidative damage, as well as inducing cardiac fibrosis via angiotensin II- and endothelin 1-induced collagen accumulation [11].

Considerable evidence verifies a strong correlation among biological age, sex, and cardiovascular risk. While the incidence and progression of CVDs are less in premenopausal women compared to age-matched men, as a consequence of age-related estrogen deficiency, this sex advantage for women decreases or disappears [12]. Although advanced age is an independent risk factor for CVDs, reduced estrogen level could further deteriorate cardiac outcomes in a female aging population [13].

In this context, we hypothesize that replacement of aging-induced estrogen loss may possess therapeutic efficacy in the mitigation of cardiac oxidative damages. The main purpose of our study is to examine the impact of hormone replacement therapy on antioxidant defense systems and cardiac remodeling in ovary-intact aged female rats.

## 2. Materials and Methods

### 2.1. Experimental Design

In our study, fertile control (*n* = 20) and 20-month-old (aging) ovary-intact female Wistar rats (*n* = 66) (Toxi-Coop Zrt., Hungary) were used and housed (Directive 2010/63/EU) under constant temperature (20–22°C) and humidity (40–50%) with a 12 h light/dark cycle. Phytoestrogen-free chow and tap water were available *ad libitum*. At the age of 20 months, aging rats were randomly assigned (10-12 rats per group) to receive either estrogen (E_2_, 0.1 mg/kg/day oral treatment, Estrofem, Novo Nordisk A/S, Bagsvaerd, Denmark) or raloxifene (RAL, 1.0 mg/kg/day oral treatment, Evista, Munich, Germany), which were calculated based on our previous study [14]. Each treatment was carried out in our laboratory by the same person. Both E_2_ and RAL administration were always performed at the same time of the day, preferably in the morning. The health status of the animals was monitored before, during, and after the treatments. In our experiment, all efforts were made to minimize the number of animals as well as the animal suffering. After 2 weeks of treatment, both control and aging rats were euthanized (100 mg/kg thiopental, B. Braun Medical SA, Barcelona, Spain) and divided for induction of ischemia/reperfusion (I/R) injury at a Langendorff perfusion apparatus or were sacrificed for biochemical measurements. For biochemical assays, heart samples were excised, nap frozen in liquid nitrogen, and stored at –80°C for further biochemical analysis. The experimental protocol and animal groups are presented in Figure 1.

The animal protocols were examined and approved by the Institutional Ethical Committee and were performed in accordance with the standards of the European Community guidelines on the care and use of laboratory animals (I.74-40/2017. MÁB).

### 2.2. Measurement of Cardiac HO Activity

Cardiac samples were homogenized in an ice-cold buffer (10.0 mM N-2-hydroxyethylpiperazine-N′-2-ethanesulfonic acid, 32.0 mM sucrose, 1.0 mM dithiothreitol (DTT), 0.10 mM ethylenediaminetetraacetic acid disodium salt dihydrate (EDTA), 10.0 *μ*g/mL trypsin inhibitor, 10.0 *μ*g/mL leupeptin, and 2.0 *μ*g/mL aprotinin; pH 7.4). After centrifugation at 15000 × *g* for 20 min at 4°C, supernatant fractions were collected. The reaction mix contained 2.0 mM glucose-6-phosphate, 0.14 U/mL glucose-6-phosphate dehydrogenase, 15.0 *μ*M hemin, 120.0 *μ*g/mL rat liver cytosol as a source of biliverdin reductase, 2.0 mM MgCl_2_ × 6H_2_O, 100.0 mM KH_2_PO_4_, and 150.0 *μ*L supernatant. The reaction was started by adding 100.0 *μ*L reduced *β*-nicotinamide adenine dinucleotide phosphate (*β*-NADPH) and incubation in the dark for 60 min at 37°C. The reaction was stopped by ice cooling. The bilirubin content was determined according to the optical density that was measured at 465 nm and 530 nm, and the difference between the two densities was calculated. HO activity was defined as the amount of bilirubin (nmol) produced per hour per mg protein [15].

### 2.3. Measurement of Cardiac Total Glutathione (GSH+GSSG) Content

To determine the cardiac GSH+GSSG content, heart samples were homogenized in a solution of 0.25 M sucrose, 1 mM DTT, and 20 mM Tris and then centrifuged at 15000 × *g* for 30 min at 4°C; then, 0.1 M CaCl_2_, 0.25 M sucrose, 20 mM Tris, and 1 mM DTT were added to the supernatants. After incubation at 0°C for 30 min, the samples were further centrifuged at 21450 × *g* for 60 min at 4°C. As a diluent buffer, a mixture of 125 mM Na phosphate and 6.0 mM EDTA was used for the stock solution of glutathione (GSH), glutathione reductase, 5,5′dithio-bis-2-nitrobenzoic acid (DTNB), and *β*-NADPH. A total volume of 40 *μ*L of each blank, standard, or heart sample and equal volumes of DTNB stock solution (20 *μ*L) and *β*-NADPH (140 *μ*L) were added to each well and then incubated at 25°C for 5 min. A 10 *μ*L volume of glutathione reductase was used to initiate the reaction, and the absorbance was measured at 405 nm.

In the spectrophotometric assay for total GSH, GSH was sequentially oxidized by DTNB and reduced by NADPH in the presence of glutathione reductase. Total glutathione values were expressed as nmol/mg protein [16].

### 2.4. Measurement of Cardiac MMP-2 Activity

Gelatin zymography was used to evaluate the MMP-2 activity in the cardiac tissue. The protein concentration was determined by the Bradford method, and then, 70 *μ*g protein was loaded to the 8% sodium dodecyl sulfate- (SDS-) polyacrylamide gel copolymerized with gelatin (20 mg/mL; type A from porcine skin; Sigma). Following electrophoresis, the gels were washed with 2.5% Triton X-100 and incubated overnight at 37°C in an incubation buffer containing 50 mM Tris-HCl, 150 mM NaCl, and 5 mM CaCl_2_. A staining method was performed by using 0.05% Coomassie Brilliant Blue, and then, a mixture of 4% methanol and 8% acetic acid was added to the gels. Following washing procedures, the gels were digitally scanned and analyzed by using Quantity One software. MMP-2 human recombinant (Sigma-Aldrich, Hungary) was used as a positive control to identify MMP-2 activities, which were expressed as intensity × mm^2^ [16].

### 2.5. Measurement of Collagen Type I and TIMP-2 Concentrations

Cardiac samples were homogenized in phosphate buffer (pH 7.4) for 20 seconds. After centrifugation (20 min, 2500 rpm, 4°C), supernatants were collected carefully and used for ELISA (GenAsia, Shanghai) and protein measurements. During ELISA measurements, blank, standard, and LV supernatants were probed by using a second antibody labeled with biotin for 60 minutes at 37°C. After washing procedures, samples were incubated with chromogen A and B solutions for 10 minutes at 37°C, and then, the reaction was stopped. Both collagen type I and TIMP-2 concentrations were determined at 450 nm and given as ng/mg protein.

### 2.6. Protein Determination

Using a commercial protein assay kit (Bio-Rad Labs), 20 *μ*L aliquots of the samples was mixed with 980 *μ*L of distilled water, and then, 200 *μ*L Bradford reagent was added to each dilution. After mixing and following 10 min incubation, the standard and sample dilutions were assayed spectrophotometrically at 595 nm. Protein levels were expressed as mg protein/mL.

### 2.7. Regional Ischemia/Reperfusion Protocol

Rat hearts were isolated, transferred to the Langendorff perfusion apparatus, and perfused with Krebs-Henseleit buffer (11.2 mM glucose, 1.24 mM KH_2_PO_4_, 20.1 mM NaHCO_3_, 119 mM NaCl, 4.7 mM KCl, 1.25 mM CaCl_2_, and 1.24 mM MgSO_4_) equilibrated with 95% O_2_ and 5% CO_2_ at 37°C. After 10 min of stabilization, regional ischemia was induced by ligation of the left anterior descending (LAD) coronary artery for 30 min, and then, reperfusion was maintained for 120 min. At the end of the reperfusion, hearts were stained with 1% Evans blue solution via the cannula. Heart samples were frozen at –20°C overnight [16].

### 2.8. Evaluation of Infarct Size

Frozen hearts were cut into 2 mm thick cross-sectional slices, which were stained with 1% 2,3,5-triphenyltetrazolium chloride (TTC) solution prepared in phosphate buffer saline (pH 7.4) and incubated for 10 min at 37°C. After TTC staining, the slices were transferred to a formalin solution for 10 min and then placed to phosphate buffer (pH 7.4). Heart slices were then placed between two sheets of glass and scanned into a computer, and infarct size was calculated as the percentage of the area at risk.

### 2.9. Statistical Analysis

The results are expressed as means ± S.E.M. After verifying the Gaussian distribution of data in the groups by means of the Shapiro-Wilk test, differences of means among the groups were compared using one-way ANOVA followed by the Tukey posttest, and *p* < 0.05 was considered to be significant.

## 3. Results

### 3.1. Measurement of Cardiac HO Activity

In our experiment, HO activity was defined as the amount of bilirubin (nmol) produced per hour per mg protein. Regarding the shift in redox status, the antioxidant HO enzyme activity significantly decreased in the myocardium of aged rats compared to the control animals. Two weeks of either E_2_ or RAL treatment enhanced the HO activity, thus indicating improvement in redox balance. Data and *p* values are presented in Figure 2.

### 3.2. Measurement of Cardiac Total Glutathione (GSH+GSSG) Content

GSH is a critical nonenzymatic antioxidant that protects the heart against oxidative damage. Our findings show that advanced age is associated with GSH depletion; nevertheless, a decreased GSH value was restored by hormone replacement therapy. While oral administration of E_2_ resulted in a ~40% increase compared to the aging group, RAL treatment elevated (~100%) the GSH content more efficiently. Data and *p* values are presented in Figure 3.

### 3.3. Measurement of Cardiac Collagen Type I Concentration

To determine the age-induced alterations in fibrotic mechanisms and to test the potential protective effects of hormone replacement therapies, cardiac collagen type I concentration was measured. Our data revealed significant remodeling in the hearts of aged rats. Aging animals displayed 9-fold higher collagen accumulation compared to the control counterparts; however, 2-week-long administration of E_2_ and RAL significantly reduced the pathological collagen content. Data and *p* values are presented in Figure 4.

### 3.4. Measurement of Cardiac MMP-2 Activity

If hormone replacement therapy exhibits protective effects on the aged hearts by modulating collagen degradation, then an effect on MMP-2 activation was expected. Our results show that the aging process resulted in a 70% decrease in the MMP-2 activity compared to the control group. In addition, both E_2_ and RAL treatments significantly increased the cardiac MMP-2 activity. Data and *p* values are presented in Figure 5(a).

### 3.5. Measurement of Cardiac TIMP-2 Concentration

To examine whether hormone replacement therapy modulates and upregulates MMP-2 activity, its tissue inhibitor was also tested. Similar to the MMP-2 activity, we found that cardiac TIMP-2 concentration was significantly reduced in the aged hearts. Data and *p* values are presented in Figure 5(b).

### 3.6. Evaluation of Infarct Size

As shown in Figure 6, a significant increase in the ratio of infarct size was observed in the aged hearts compared to the control group. Again, administration of E_2_ or RAL replacement resulted in a significant decrease compared to the aging counterparts, suggesting the protective effects of hormone replacement therapy on myocardial I/R injury. The mean values of the area at risk (AAR) are as follows: control: 41.99, aging: 43.56, aging+E_2_: 39.48, and aging+RAL: 42.95.

## 4. Discussion

With a keen awareness that aging is an independent risk factor for CVDs, a better understanding of the potential biological mechanisms underlying cardiovascular aging and pursuits to decrease the risk of CVDs are necessary to improve the quality of life for the elderly. Epidemiological data verify the sex advantage of premenopausal women against CVDs; however, this favorable property becomes far less or disappears with advanced age due to reduced estrogen level [12, 17]. Under physiological conditions, estrogen possesses antioxidant effects, attenuates inflammation, and induces angiogenesis as well as vasorelaxation that protect the heart against molecular and functional injuries [10]. Nevertheless, the estrogen-mediated cardioprotective effects are reduced during aging due to the fluctuation of 17*β*-estradiol level, which is the most potent estrogen during the premenopausal period. The reduction of estrogen synthesis, changes in estrogen receptors, and alterations of signaling pathways related to the aging process increase the risk of complex cardiovascular damages [18].

The use of hormone replacement therapy (HRT) is still controversial. The reason for the different characterization of HRT includes many factors that contribute to the various outcomes, among them the duration and dosage of the hormone administration [19, 20]. While most research studies focus on the ovariectomy-induced estrogen depletion, less information is available on the age-related response to hormone replacement therapy. Therefore, our experimental protocol was designed to evaluate the hypothesis that HRT may be a potential therapeutic strategy to achieve successful aging via reducing cardiac risk factors. Our findings show that age-induced decrease in estrogen level (control: 287.91 ± 6.73 ng/L, aging: 171.77 ± 7.00 ng/L) reflected on the measured *ex vivo* and biochemical parameters via altering the redox status and inducing abnormal cardiac remodeling; however, 2 weeks of HRT (estrogen or raloxifene) was able to restore the adverse effects.

As it is well known, oxidative damage occurs as a result of the failure in antioxidant mechanisms to eliminate ROS production. Numerous studies verify that HO is a key molecule against oxidative injuries through its antioxidant and anti-inflammatory properties [21–23]. The HO isoforms (HO-1, HO-2, and HO-3) are known to catalyse the oxidation of heme to generate free iron, CO, and biliverdin, which is subsequently reduced to bilirubin by biliverdin reductase. Both biliverdin and bilirubin possess antioxidant capacity, while CO is a vasodilator and anti-inflammatory and antiapoptotic molecule [24, 25]. In our study, we detected that the aging process significantly reduced the HO enzyme activity compared to the control/fertile group, which suggests that cells became more vulnerable to oxidative insult. In a previous study, Ungvari et al. investigated the role of a nuclear factor erythroid-2 related factor-2 (Nrf2) redox-sensitive transcriptional regulator in cardiovascular aging [26]. During physiological conditions, Nrf2 leads to the upregulation of various antioxidant genes, such as HO-1; however, age-related ROS production fails to activate Nrf2, resulting in oxidative damage and inflammation. In another study, Kwon et al. evaluated the effect of the Nrf2/HO-1 signaling pathway on antioxidant capacity [27]. Their results showed that Nrf2/HO-1 signaling resulted in an enhancement of GSH content, whereas inhibition of the HO-1 activity eliminated the cytoprotective effect of GSH. In our work, the aging process caused a similar reduction in both HO activity and GSH content, which suggests that these antioxidant mechanisms may be mediated through Nrf2 signaling. While aging/estrogen deficiency was associated with shift in the redox status, estrogen and raloxifene treatments exert protective effects on the cardiac antioxidant status via increasing HO activity and GSH level. These results are in accordance with our earlier observations, where the antioxidative role of estrogen and raloxifene was verified in ovariectomized rat models [14]. Raloxifene is a selective estrogen receptor modulator (SERM), which acts either as an estrogen agonist or as an antagonist in a tissue-selective manner. This benzothiophen derivate binds with high affinity to the nuclear estrogen receptor; thus, its pharmacological profile is similar to that of estrogen, particularly in the cardiac tissue [28]. Konyalioglu et al. reported that 1 mg/kg raloxifene treatment caused a significant elevation in the cardiac GSH level of ovariectomized rats [29]. Reduction of GSH due to ovariectomy-induced estrogen loss or the aging process is due to a yield of ROS overproduction, which promotes oxidative damage and inflammatory processes.

Considerable evidence has been published that cardiac senescence is associated with mitochondrial dysfunction, mitochondrial DNA mutations, and oxidative damage to respiratory enzymes, which result in a significant increase in ROS [30]. In agreement with the beneficial role of estrogen on the heart, estrogen receptors localized on the mitochondrial membrane are significant elements of estrogen-mediated cell survival and cardioprotection. Previous studies proved that activation of mitochondrial ER*α*, ER*β*, and GPR30 receptors protects against ex vivo I/R injury, results in a smaller infarct size, and possesses an ROS scavenging role [31].

Given the complexity of age-mediated ROS accumulation and disruption of antioxidant defense mechanisms, the heart is especially prone to oxidative damage and morphological and functional alterations. Therefore, aging is considered a predisposing factor for cardiac fibrosis, which is characterized by decreased myocyte number, increased myocyte size, and accumulation of the extracellular matrix (ECM), especially the collagen [32]. Myocardial ECM is essential for proper cardiac structural integrity and pump function and possesses a mediator role in the modulation of the cardiac phenotype during hypertrophy [33]. ECM depends on a well-controlled balance between the matrix metalloproteinases (MMPs) and the tissue inhibitor of metalloproteinases (TIMPs). MMPs are Ca^2+^ and Zn^2+^-dependent proteases that are synthesized as inactive forms or pro-MMP and can be activated by removal of an amino-terminal propeptide domain. Among the 26 MMPs, MMP-2 is involved in cardiac remodeling via cleaving collagen type I and type III. Although activated MMPs intensively degrade the ECM proteins, their endogenous inhibitors, namely, TIMPs, have a compensatory role to prevent excessive ECM degradation [34]. Therefore, the balance between MMPs and TIMPs determines the synthesis and degradation of cardiac ECM. During aging, the ECM remodeling is disrupted, which induces excessive collagen accumulation in the heart (i.e., fibrosis) [35]. Our data prove that the aging process increases the cardiac collagen content via disrupting the MMP-2/TIMP balance. We found that collagen type I concentration significantly increased in aged hearts compared to the control/fertile counterparts. Consistent with Kwak et al., we noted that age-associated collagen deposition is a consequence of cellular events including increased collagen synthesis and decreased degradation, which resulted from the disruption of MMP-2/TIMP signaling [36]. Our hypothesis whether hormone replacement therapy plays a beneficial role in the cardiac remodeling was underpinned with the reduced collagen level and the elevated MMP-2/TIMP values. Similar to our findings, Mountain et al. demonstrated a significant reduction in MMP-2 and TIMP-2 levels in response to ovariectomy; however, hormone replacement therapy resulted in the upregulation of MMP-2, indicating that hormone substitution modulated the MMP-2 regulatory pathway [37]. In another research work, Xu et al. supported the antifibrotic effects of estrogen in the prevention of left ventricular remodeling [38]. Estrogen replacement therapy was indicated to reduce left ventricular weight and collagen accumulation in 12-month-old ovariectomized rats, via enhancing MMP-2 activity. Furthermore, they verified that aging-mediated collagen accumulation and the decreased MMP-2 activity were associated with the downregulation of ER*α* and ER*β*.

Besides antioxidative and anti-inflammatory properties, numerous studies indicate in different models that HO possesses a favorable impact on cardiac remodeling. Wang et al. established that the upregulation of HO-1 promoted neovascularization and limited oxidative stress, myofiber hypertrophy, and interstitial fibrosis, which were associated with improved chamber remodeling and systolic/diastolic function [8]. Further finding supported the beneficial role of HO in the attenuation of cellular senescence during the development of myocardial infarction in an aged heart [39].

In view of the importance that HO serves as a defense mechanism against oxidative stress and in cardiac remodeling, we investigated its potential role in I/R injury in aged rats. Accumulating data showed that the HO/CO pathway is a potential defense line against I/R injury [39, 40]. Upon the release of CO, it activates the enzyme soluble guanylate cyclase (sGC) and induces vasorelaxation by increasing cyclic guanosine monophosphate (cGMP). Studies with ovariectomized rats supported that excessive generation of ROS promoted oxidative damage and inflammation and impaired the sensitivity for cardiac ischemia, although hormone replacement seemed to be an effective therapy in the mitigation of adverse effects [13, 14]. Similar to these observations, our results clearly show that both estrogen and raloxifene substitution significantly decreased the ischemic ratio after LAD occlusion, which may be consequently associated with the upregulation of the HO system in aged rats.

In our present study, we gained insights into age-related disturbances in oxidant/antioxidant homeostasis and adverse fibrotic mechanisms. A better understanding of the molecular and cellular mechanisms underlying cardiovascular aging provides potential targets for specific interventions to delay or prevent pathological cardiac processes. Our findings show that both estrogen and raloxifene replacements restored antioxidant defense systems and reduced the excessive collagen accumulation via enhancing the MMP-2/TIMP-2 signaling mechanism. The increase in HO activity and GSH content as well as the improvement in fibrotic processes could reduce I/R-induced necrotic ratio. In this sense, we can conclude that 2-week-long low-dose estrogen or raloxifene replacement therapy seems to be an efficient approach to promote successful cardiovascular aging.

## Figures and Tables

**Figure 1:** The experimental protocol of the study. E_2_: estrogen; RAL: raloxifene; HO: heme oxygenase; GSH: glutathione; MMP-2: matrix metalloproteinase-2; TIMP-2: tissue inhibitor of matrix metalloproteinase-2.

**Figure 2:** The effects of the aging process and E_2_/RAL treatment on cardiac HO activity (HO, expressed as nmol bilirubin/h/mg protein). Result shown as means ± S.E.M. *n* = 9–10. ^∗^*p* < 0.05: statistical significance relative to the control group. ^#^*p* < 0.05: statistical significance relative to the aging group. E_2_: estrogen; RAL: raloxifene.

**Figure 3:** The effects of the aging process and E_2_/RAL treatment on cardiac GSH+GSSG content (GSH+GSSG, expressed as nmol/mg protein). Result shown as means ± S.E.M. *n* = 9–10. ^∗^*p* < 0.05: statistical significance relative to the control group. ^#^*p* < 0.05: statistical significance relative to the aging group. E_2_: estrogen; RAL: raloxifene.

**Figure 4:** The effects of the aging process and E_2_/RAL treatment on cardiac collagen type I content (expressed as ng/mg protein). Result shown as means ± S.E.M. *n* = 8–9. ^∗^*p* < 0.05: statistical significance relative to the control group. ^#^*p* < 0.05: statistical significance relative to the aging group. E_2_: estrogen; RAL: raloxifene.

**Figure 5:** (a) The effects of the aging process and E_2_/RAL treatment on cardiac MMP-2 activity (64 kDa MMP-2, expressed as intensity∗mm^2^). Result shown as means ± S.E.M. *n* = 8–10. ^∗^*p* < 0.05: statistical significance relative to the control group. ^#^*p* < 0.05: statistical significance relative to the aging group. E_2_: estrogen; RAL: raloxifene. (b) The effects of the aging process and E_2_/RAL treatment on cardiac TIMP-2 concentration (TIMP-2, expressed as ng/mg protein). Result shown as means ± S.E.M. *n* = 7–9. ^∗^*p* < 0.05: statistical significance relative to the control group. ^#^*p* < 0.05: statistical significance relative to the aging group. E_2_: estrogen; RAL: raloxifene.

**Figure 6:** The effects of the aging process and E_2_/RAL treatment on the ratio of infarct size (IS/AAR, expressed as %). Result shown as means ± S.E.M. *n* = 9–11. ^∗^*p* < 0.05: statistical significance relative to the control group. ^#^*p* < 0.05: statistical significance relative to the aging group. E_2_: estrogen; RAL: raloxifene; IS: infarct size; AAR: area at risk.

## Data Availability

Each necessary result, data, and statistics is presented through the manuscript.
